# Long Noncoding RNA TUG1 Aggravates Cerebral Ischemia/Reperfusion Injury by Acting as a ceRNA for miR-3072-3p to Target St8sia2

**DOI:** 10.1155/2022/9381203

**Published:** 2022-04-19

**Authors:** Miao Chen, Feng Wang, Limin Fan, Hairong Wang, Shuo Gu

**Affiliations:** ^1^Department of Emergency, The First Affiliated Hospital of Hainan Medical University, No. 31, Longhua Road, Longhua District, Haikou City, Hainan Province 570102, China; ^2^Neurology Department, Seventh People's Hospital of Shanghai University of Traditional Chinese Medicine, Shanghai 200137, China; ^3^The Institute for Biomedical Engineering and Nano Science, Tongji University School of Medicine, No. 1239, Siping Road, Shanghai 200092, China; ^4^Department of Emergency, Xinhua Hospital Affiliated to Shanghai Jiaotong University, School of Medicine, No. 1665, Kongjiang Road, Shanghai 20092, China; ^5^Department of Pediatric Neurosurgery, The First Affiliated Hospital of Hainan Medical University, No. 31, Longhua Road, Longhua District, Haikou City, Hainan Province 570102, China

## Abstract

Long noncoding RNA taurine-upregulated gene 1 (TUG1) is considered to be involved in postischemic cerebral inflammation, whereas polysialic acid (polySia, PSA), the product of St8sia2, constitutes polysialylated neural adhesion cell molecule (PSA-NCAM) in both mice and humans and that cerebral PSA-NCAM level is elevated in neuronal progenitor cells in response to transient focal ischemia. Herein, we aim to identify novel miRNAs that bridge the functions of St8sia2 and TUG1 in ischemia-associated injuries. In both *in vivo* (C57BL/6J mouse ischemia/reperfusion, I/R model) and *in vitro* (mouse neuroblastoma N2A cell oxygen glucose deprivation/reoxygenation, OGD model) settings, we observed upregulated TUG1 and St8sia2 after the induction of ischemic injury, accompanied by reduced miR-3072-3p expression. We performed siRNA-induced TUG1 knockdown combined with the induction of ischemic injury; the results showed that inhibiting TUG1 expression led to the reduced infarct area and improved neurological deficit. Through bioinformatics analysis, miR-3072-3p was found to target both St8sia2 and TUG1, which was subsequently verified by the luciferase reporter system and RNA binding protein immunoprecipitation assay. Also, the addition of miR-3072-3p mimic/inhibitor resulted in reduced/elevated St8sia2 expression at the protein level. Further studies revealed that in both *in vivo* and *in vitro* settings, TUG1 bound competitively to miR-3072-3p to regulate St8sia2 expression and promote apoptosis. In summary, targeting the TUG1/miR-3072-3p/St8sia2 regulatory cascade, a novel cascade we identified in cerebral ischemia injury, may render feasible therapeutic possibilities for overcoming cerebral ischemic insults.

## 1. Introduction

Stroke is also called cerebral infarction. In the past four decades, the prevalence of stroke has declined by 42% in high-income countries and doubled in low-income countries [1]. In China, the annual new cases of stroke are up to 2 million, with an upward trend of stroke incidence among the young population [2], and more than 65% of the surviving patients have different degrees of disability [3]. The direct medical expenses for stroke care in China increased rapidly at an average annual growth rate of 18.04%, reaching 37.45 billion yuan in 2003, accounting for 6.52% and 5.68% of the total medical and health expenses, respectively [4]. Therefore, stroke poses a serious threat to the health of the population and brings a heavy economic burden to the society.

Thrombolytic drugs can be used to dissolve the newly formed “blood clots” to reopen the blood vessels and restore the blood flow, which is currently recognized as the most effective way to save the uninfarcted ischemic brain tissue [5]. However, the thrombolysis rate of acute ischemic stroke (AIS) is only 2.4% in China [6]. Although patients generally experience improvement in symptom manifested by significantly reduced or even completed restored neurological deficit at the beginning of thrombolytic drugs application, the symptoms might be aggravated again shortly afterwards, presumably related to the ischemia-reperfusion injury [7]. Therefore, further understanding of the mechanism underlying ischemia-reperfusion is crucial for better clinical outcome of ischemia.

Noncoding RNAs (ncRNAs) have been well documented to be strongly linked to stroke and poststroke recovery of neurofunction [8]; among which long noncoding RNAs (lncRNAs) as well as microRNAs (miRNAs) are the most representative ones [9, 10]. lncRNAs are a type of RNA longer than 200 nt [11] and mainly distributed in the nucleus or cytoplasm [12], with an organ- and tissue-specific expression pattern [13]. Generally, lncRNAs are transcribed by RNA polymerase II and usually undergo a splicing process, although they possess both cap structure and a polyA tail. The lack of an open reading frame (ORF) prevents them from encoding protein [14]. In recent years, lncRNAs were found to be related to multiple biological processes such as among others, X chromosome silencing [15], chromosome modification [16], transcription activation and suppression [17], cell differentiation [18], carcinogenesis [19], and ontogeny [20]. Therefore, the identification of functional lncRNAs, especially the study of the effect mechanism, has attracted more and more attention from scholars at home and abroad [21]. Several studies have indicated that lncRNAs play role in many pathophysiological processes, such as nervous system development [22], stroke [23], and Alzheimer's disease [24]. Taurine-upregulated gene 1 (TUG1) is a highly conserved member of the lncRNA family and widely expressed throughout the body tissues. Previous studies indicated that THG1 was indispensable for male fertility [25] and involved in the progression of preeclampsia [26]. Importantly, TUG1 was found to be a sponge of miR-145a-5p, thus modulating microglial polarization of BV-2 microglial cells that undergo glucose deprivation [27], indicating its pivotal role in cerebral inflammation. Moreover, another study on myocardial infarction revealed a potential TUG1-miR-9a-5p axis that mediates apoptosis of cardiomyocyte [27]. Hence, we hypothesized that TUG1 might also be involved in the ischemia stroke.

Sialyltransferase 2 (St8sia2) is a polysialyltransferase [28]. A recent research has found that St8sia2 is related to the remodeling of nerve cells and the interaction between neurons [29]. It is also closely related to Alzheimer's disease [30], anxiety [31], and manic depression [32]. Of note, a previous study on human brain ischemia showed that the combination of polysialic acid (polySia, PSA, the main product of St8sia2) moiety and neural adhesion cell molecule (NCAM), abbreviated as PSA-NCAM, was significantly elevated in neuronal progenitor cells (NPCs) [33], implying the involvement of St8sia2 in this process. However, the direct relationship between St8sia2 and stroke has not yet been reported so far.

Considering that both TUG1 and St8sia2 are associated with ischemia stroke, this paper is aimed at elucidating the way through which they work in concert to regulate the ischemic process. In addition, there have been no reports on the correlation of TUG1 and St8sia2 in any other field; thus, the novelty and motivation of the study are to first identify the relationship between TUG1 and St8sia2 in cerebral ischemia/reperfusion injury. Besides, miRNA is an important member of the ncRNA family. Past evidence has indicated that miRNAs exert a negative regulatory function mainly by binding to their target genes' mRNA and promoting mRNA degradation/inhibiting mRNA translation [34]. Recent studies have found that miRNAs have a wide range of effects on stroke [35]. The miRNAs unique to brain tissues participate in the regulation of different physiological and pathological processes of the nervous system, such as the occurrence, development, synapse formation, and neuroprotection of the nervous system [36], aside from their involvement in cerebral infarction, cerebral hemorrhage, brain trauma, Parkinson's disease, and cognitive impairment [37]. Given the foregoing, we assumed that miRNA might bring TUG1 and St8sia2 together to regulate the ischemia-associated pathological processes. To verify the joint action of TUG1, St8sia2, and miRNA in ischemia stroke, a series of experiments was performed in the current study; the corresponding effects on ischemia-reperfusion injury were also investigated.

## 2. Material and Methods

### 2.1. Rat Ischemia/Reperfusion (I/R) Model

All animal experiments had got ethical approval from the University of Shanghai for Science and Technology and were conducted strictly following the guidelines stipulated in the Institutional Animal Care and Use. The experimental animals were male C57BL/6J mice (6–8 weeks of age, 25 ± 5 g) supplied by the Shanghai SLAC Laboratory Animal Co., Ltd. (Shanghai, China). Following previously reported procedures, intraluminal middle cerebral artery occlusion (MCAO) [38] was performed to establish focal cerebral ischemia, followed by reperfusion 2 h later. Under isoflurane anesthetization, mice were placed on a heating panel kept at 37.0°C ± 0.5°C throughout the procedure. Animals after 24 h of reperfusion were reared for an additional two weeks and then euthanized. The same surgical procedure was performed on sham-operated mice in the absence of MCAO.

### 2.2. Infarct Area Determination

2,3,5-Triphenyltetrazolium chloride monohydrate (TTC; Sigma-Aldrich) staining was performed to identify the brain infarct area 48 h post-MCAO treatment. In brief, 2 min thick coronal brain slices were immobilized overnight in 10% formaldehyde after 15 min of soaking in 2% TTC solution. After observing the caudal and rostral surfaces of each slice, the percentage of infarct area was computed with the use of ImageJ software (NIH, USA).

### 2.3. Evaluation of Neurological Deficits

Referring to a previous neurological deficit score [39], mice were scored for neurological status 24 h postreperfusion with the criteria described as follows: 0: absence of observable deficits; 1: difficulty in fully extending the contralateral forelimb; 2: inability to extend the contralateral forelimb; 3: slight circling to the contralateral side; 4: severe circling to the unaffected side; 5: falling to the unaffected side. The evaluation and grading of the animals were made by a scientist who had no knowledge of treatments.

### 2.4. Terminal Transferase Uridyl Nick End Labeling (TUNEL) Assay

Apoptosis, as manifested by severely damaged DNA, was assessed by TUNEL staining. N2A as well as mouse brain tissue staining was performed using either the ApopTag Kit S7100 (Millipore, Temecula, CA, USA) or TUNEL Apoptosis Detection Kit (Abbkine Scientific, Waltham, MA, USA) following the supplier's recommendations, whereas the cell nucleus was counterstained with DAPI. A Nikon ECLIPSE Ti confocal microscope (×200 magnification) was utilized for the calculation of TUNEL-positive cell nuclei. The percentage of TUNEL-positive cell nuclei in 10 randomly selected fields was used to calculate the apoptosis (%) in each sample.

### 2.5. Immunohistochemistry Analysis

The brain tissues that underwent I/R or sham operation were subjected to 24 h of paraformaldehyde (4%) immobilization and paraffin embedding before being sliced into sections (5 *μ*m thickness). The prepared sections underwent subsequent dewaxing and antigen repair; the endogenous antigen was then inactivated by hydrogen peroxide. They were then treated with 3 PBS washes and 30 min of culture in 5% bovine serum albumen (BSA) prior to incubation (4°C) with St8sia2-specific polyclonal antibody (Proteintech Group, Rosemont, IL, USA). 24 h postincubation, the resultant reactions were visualized by staining with horseradish peroxidase and diaminobenzidine. St8sia2 expression was evaluated based on IHC images using ImageJ software.

### 2.6. Stereotaxic Injection

After anesthesia, the mice were fixed to a stereotaxic apparatus supplied by David Kopf Instruments, Tujunga, CA, USA. Then, a mixture prepared by si-TUG1/miR-3072-3p-mimic/si-St8sia2 (5 *μ*l) or corresponding scrambled controls (109 infectious units/ml; GenePharma, Shanghai, China) with *in vivo* RNAiMAX transfection reagent (Invitrogen) was administered via mouse lateral ventricle. MCAO was performed 24 h later. 0.2 mm posterior to bregma, 1.0 mm lateral to the midline, and 1.5 mm below the brain surface were used as stereotaxic coordinates.

### 2.7. Cell Cultivation and Oxygen Glucose Deprivation/Reoxygenation (OGD/R) Model [40]

In a humidified incubator at 37°C with 5% CO_2_ in air, mouse neuroblastoma cells (N2A; Cell Bank of Shanghai Institute of Cell Biology, Chinese Academy of Sciences, Shanghai, China) were cultivated in Dulbecco's Modified Eagle's Medium (DMEM; Invitrogen) added with 10% fetal bovine serum (FBS; Invitrogen) +2 mM glutamine (Invitrogen) + 100 *μ*g/ml streptomycin (Invitrogen) + 100 U/ml penicillin (Invitrogen). To investigate the impacts of ischemia *in vitro*, the cells underwent OGD treatment by 4 h of incubation (37°C) with opti-MEM (Invitrogen) in a hypoxic chamber with 5% CO_2_ and 95% N_2_ in air. The cells were then immersed in a normal culture medium and kept under normoxia (5% CO_2_, 37°C) for 24 h.

### 2.8. Construction of Plasmid Cloning Vehicles and Transfection of Cells

For TUG1 overexpression, pcDNA3.1-TUG1 plasmids were constructed via subcloning the mouse full-length TUG1 cDNA into the pcDNA3.1(+) mammalian expression vector (Invitrogen) at the KpnI and XhoI loci. DNA Midiprep kits (Qiagen, Germany) were employed for the isolation of all plasmids. N2A cells post pcDNA3.1-TUG1 transfection were collected using G418 (geneticin) to produce stable clones. Those with empty pcDNA3.1(+) vector (pcDNA3.1-NC) transfection functioned as negative control. As to miR-3072-3p overexpression and knockdown, the synthesis of miR-3072-3p mimic and inhibitor, along with two scrambled miRNAs that served as their corresponding negative controls (mimic-NC and inhibitor-NC for miR-3072-3p mimic and miR-3072-3p inhibitor, respectively), was done at Qiagen (Germany). For all transfections, Lipofectamine 3000 reagent (Invitrogen) was used following the recommendations.

### 2.9. qPCR Analysis

The TRIzol (Invitrogen)-isolated total RNA from cell samples was quantified before being reversely transcribed. Reverse transcription reactions of RNA/miRNA were performed by PrimeScript™ RT Master Mix and SYBR® PrimeScript™ miRNA RT-PCR kit, respectively, both supplied by TaKaRa (Shiga, Japan). The primer sequences are shown in Table 1. According to the manufacturer's protocol, rapid real-time polymerase chain reaction (QPCR) and FastStart Essential DNA Green Master (Rosh, Indiana, USA) were employed for the determination of the levels of reverse-transcribed cDNA templates relative to *β*-actin. Each test was run in triplicate, and fold changes were computed by 2^-∆∆CT^, a relative quantification method. The device used for amplification tests was ROCHE 480II real-time PCR machine (ROCHE, USA).

### 2.10. Western Blot

Cells after cultivation were collected and lysed in RIPA lysis buffer (P0013B; Beyotime, Shanghai, China) after ice-cold PBS washing. After detecting the protein concentration using the BCA protein assay kit (P0012; Beyotime), the whole lysates were immersed in a 5x SDS loading buffer (P0015; Beyotime) at 1 : 4. Then, samples with equal amounts were subjected to isolation by sodium dodecyl sulfate (SDS) polyacrylamide gel electrophoresis (PAGE) and subsequent transfer onto PVDF membranes at 180 mA for 60 min. Blots were blocked for 2 h in TBST added with 5% skim milk and then cultivated (4°C) overnight with *Ι* antibodies. This was followed by treatment with horseradish peroxidase- (HRP-) labeled (1 : 1000, Cell Signaling Technology, USA) secondary antibodies. The *Ι* antibodies were anti-Bcl2 (1 : 1000, Cell Signaling Technology, USA), anti-Bax (1 : 1000, Cell Signaling Technology, USA), and anti-St8sia2 (1 : 200, Proteintech, USA). *β*-Actin (1 : 1000, Cell Signaling Technology, USA) was the internal control. The protein expression was normalized to *β*-actin. Chemiluminescence was performed with an enhanced chemiluminescence detection kit to display protein bands according to the manufacturer's recommendations.

### 2.11. Luciferase Reporter Gene Assay (LRGA)

By using StarBase and TargetScan with URLs of http://starbase.sysu.edu.cn/mirMrna.php and http://www.targetscan.org, respectively, putative miR-3072-3p binding sites in both the sequence of TUG1 and the 3′-UTR of St8sia2 were predicted. Genechem (Shanghai, China) was responsible for the synthesis of the wild-type (WT)/mutant (MUT) TUG1 sequence and the WT/MUT 3′-UTR fragment of St8sia2 containing putative miR-3072-3p binding sites and then came the cloning of the synthesized sequences into pmirGLO dual luciferase reporter vector (Promega, Madison, WI, USA) downstream to generate TUG1-WT/MUT as well as St8sia2-WT/MUT luciferase reporter systems. Thereafter, N2A cells seeded onto 24-well plates were treated with luciferase reporter plasmids, miR-3072-3p mimic and its nonspecific control mimic-NC, as well as miR-3072-3p inhibitor and its nonspecific control inhibitor-NC transfections for 48 h, either alone or in combination. The Dual LRGA system (Promega, Madison, WI, USA) was utilized for luciferase activity determination, and the data were normalized to a Renilla luciferase internal control.

### 2.12. RNA Immunoprecipitation Assay

RNA-IP was performed using a RIP Kit (Millipore, Billerica, MA, USA) following the manufacturer's protocol. After being transfected miR-3072 mimic or miR-NC, N2A cells were lysed in RNA immunoprecipitation (RIP) lysis buffer and magnetic beads conjugated to human anti-Ago2 antibody (Millipore) or control IgG antibody. Then, the samples were digested with proteinase K, and RNA was extracted from the beads using TRIzol. Then, qRT-PCR analysis was performed to measure the enrichment of the miR-3072 and St8sia2.

### 2.13. Statistical Analysis

We used GraphPad Prism 8.0 (GraphPad Software, Inc., USA) to conduct statistical analyses. All data were exhibited as mean ± standard error of the mean (SEM). The intergroup and multigroup comparison was made by Student's *t*-test and one-way analysis of variance (ANOVA) with Duncan's test, respectively, with the difference considered significant when *P* < 0.05.

## 3. Result

### 3.1. In Vitro and In Vivo Ischemic Injuries Induced Upregulation of TUG1 and St8sia2 and Reduced miR-3072-3p Level

C57BL/6J mice that underwent I/R (1.5 h/24 h) exhibited obvious nerve dysfunction and serious brain infarction (Figures 1(a)–1(c)), accompanied by elevated TUG1 and St8sia2 and reduced miR-3072-3p expression at the mRNA level (Figures 1(d)–1(f)). The ischemic injury was manifested by reduced Bax/Bcl-2 ratio in both *in vivo* and *in vitro* settings (Figures 1(g) and 1(h)). Consistent with the findings by western blot, TUNEL assay revealed an increased number of apoptotic N2A cells after OGD/R treatment (Figures 1(i) and 1(j)). The alterations of TUG1, miR-3072-3p, and St8sia2 in N2A cells undergoing OGD/R treatment were similar to those in the I/R mouse model (Figures 1(k)–1(m)). These findings suggested that TUG1, miR-3072-3p, and St8sia2 might orchestrate the ischemic process.

### 3.2. TUG1 Knockdown Attenuated In Vivo Ischemic Injuries, Accompanied by Reduced St8sia2 and Elevated miR-3072-3p Levels

Since we have confirmed that TUG1 was upregulated in response to ischemic injury, to further understand the regulatory role of TUG1 in this process, we performed siRNA-induced TUG1 knockdown combined with the induction of ischemic injury, as shown in (Figures 2(a)–2(d)); inhibited TUG1 expression led to the reduced infarct area and improved neurological deficit. These improvements were coincided with reduced St8sia2 and elevated miR-3072-3p expression at the mRNA level (Figures 2(e) and 2(f)). At the protein level, the reduced Bax/Bcl-2 ratio and St8sia2 expression (Figures 2(g) and 2(h)) were observed in mice undergoing TUG1 knockdown combined with I/R treatment by comparing their siNC+I/R treatment counterparts. Consistently, the TUNEL assay (Figures 2(h) and 2(i)) showed that the absence of TUG1 attenuated the apoptosis of brain tissue that underwent I/R, which coincided with reduced St8sia2 expression as revealed by IHC (Figures 2(k) and 2(l)).

### 3.3. Forced Overexpression of TUG1 Resulted in an Ischemic-Vulnerable Phenotype of N2A Cells Opposite to That Induced by TUG1 Knockdown

To further confirm the regulatory role of TUG1 in ischemic injury, we constructed a TUG1 overexpression cell model, namely, pcDNA 3.1-TUG1-N2A cells, to perform a comparison with the effect of si-TUG1 in an *in vitro* setting. As shown in (Figure 3(a)), both overexpression and knockdown of TUG1 were successful in N2A, and miR-3072-3p/St8sia2 in mRNA level was inversely/positively correlated to the modified TUG1 expression (Figures 3(b) and 3(c)). The change of St8sia2 at the protein level in response to altered TUG1 was consistent with that in the mRNA level (Figure 3(d)), while the increased/decreased Bax/Bcl ratio was induced by TUG1 overexpression/knockdown (Figure 3(g)), suggesting that TUG1 have a proapoptotic effect, which was also verified by TUNEL assay (Figures 3(e) and 3(f)).

### 3.4. miR-3072-3p Directly Binds to St8sia2 and Regulates St8sia2 Expression

TargetScan (http://www.targetscan.org) website revealed a binding site between St8sia2 and miR-3072-3p (Figure 4(a)). To test this hypothesis, we first verified the interaction between St8sia2 and miR-3072-3p in the N2A cell model. As indicated by LRGAs, St8sia2-WT vector+miR-3072-3p mimic cotransfection significantly reduced the relative luminescence, whereas the addition of miR-3072-3p inhibitor induced an inverse trend and that no significant alteration regarding luminescence was observed in the St8sia2-MUT group (Figures 4(b) and 4(c)). The physical association between miR-3072 and St8sia2 was further confirmed by RIP analysis (Figure 4(d)). Moreover, as depicted in Figures 4(e) and 4(f), St8sia2 had an inverse connection with miR-3072-3p, further corroborating their interaction.

### 3.5. miR-3072-3p Overexpression Protects from I/R-Induced Ischemic Injury in Brain Tissues

As aforementioned, miR-3072-3p was downregulated in I/R-treated mouse brains; to better understand its role in ischemic injury, the reduced miR-3072-3p was reversed by the addition of exogenous miR-3072-3p mimic. As shown in Figures 5(a)–5(c), partial relief of I/R-induced ischemic injury was observed in the presence of miR-3072-3p mimic. In both I/R-treated and sham-operated groups, miR-3072-3p mimic effectively elevated miR-3072-3p expression (Figure 5(d)) and inhibited St8sia2 at both mRNA and protein (Figures 5(e) and 5(f)) levels, together with reduced Bax/Bcl2 ratio (Figure 5(g)) and attenuated apoptosis (Figures 5(h) and 5(i)).

### 3.6. miR-3072-3p Overexpression Protects against OGD/R-Induced Ischemic Injury in N2A Cells

For the purpose of further validating the protective action of miR-3072-3p in an *in vitro* setting, we performed both overexpression and inhibition of miR-3072 in N2A cells; as shown in Figure 6(a), the treatments of miR-3072-3p mimic and inhibitor achieved the desired results. The addition of miR-3072-3p mimic/inhibitor resulted in reduced/elevated St8sia2 expression at the protein level (Figures 6(b)–6(d)) and was responsible for attenuated/aggravated apoptosis in N2A cells (Figures 6(e)–6(g)).

### 3.7. TUG1 Acts as a ceRNA of miR-3072-3p Targeting St8sia2

Combined with the above results, we speculate that there exists a potential TUG1/miR-3072-3p/St8sia2 axis in the regulation of ischemic stroke in the cerebral hemisphere. Recognizing that miR-3072-3p could directly bind to St8sia2, we focused on the connection between TUG1 and miR-3072-3p. After StarBase prediction of the putative binding site of miR-3072-3p in TUG1 (Figure 7(a)), LRGAs were performed for confirmation. First, the interaction between miR-3072-3p and TUG1 was confirmed in Figure 7(b), where luminescence of the TUG1-WT group cotransfected with miR-3072-3p was significantly reduced, indicating that the miR-3072-3p could directly bind to TUG1; next, the indirect interaction between TUG1 and St8sia2 was confirmed in Figures 7(c) and 7(d), where overexpressed/inhibited TUG1 significantly increased/decreased the relative luminescence of the St8sia2-WT group, indicating that TUG1 might function as a ceRNA to modulate St8sia2. Finally, a TUG1-miR-3072-3p-St8sia2 regulatory axis was confirmed.

### 3.8. St8sia2 Might Account for the Regulatory Effects of the TUG1-miR-3072-3p-St8sia2 Axis in Both In Vivo and In Vitro Settings

Since proteins were responsible for the majority of biological processes [41], we speculated that the TUG1-miR-3072-3p-St8sia2 axis might converge on St8sia2. To test this hypothesis, we performed St8sia2 knockdown in both *in vivo* and *in vitro* settings. As shown in Figures 8(a)–8(c), St8sia2 knockdown significantly alleviated the I/R-induced *in vivo* ischemic injury, which might be ascribed to the high inhibitory efficiency of si-St8sia that significantly reduced the St8sia2 expression in response to I/R treatment (Figure 8(d)). Next, we detected the expression of St8sia2 and apoptosis markers in I/R-treated mouse brains; as shown in (Figure 8(e)), si-St8sia significantly reversed the I/R-induced elevation of St8sia2 level in mouse brains, accompanied by reduced Bax/Bcl2 ratio (Figure 8(f)); similar trends were observed in N2A *in vitro* cell model (Figures 8(g) and 8(h)). The si-St8sia2-mediated attenuation of apoptosis was further confirmed by TUNEL assay *in vitro* (Figures 8(i) and 8(j)) and *in vivo* (Figures 8(k) and 8(l)).

## 4. Discussion

Aberrant lncRNA expression was observed in stroke; in a previous study, thousands of differentially expressed lncRNA in patients who underwent ischemic stroke were detected by high-throughput method based on peripheral blood [42]. Several lncRNAs were related to specific ischemic processes, including inflammation and cell death induced by ischemic injury and angiogenesis that are responsible for postischemic repair and regeneration [43]. Hence, lncRNAs might serve as diagnostic markers or therapeutic target for alleviating ischemic symptoms. Altered miRNA profile was also reported in both animal stroke models and stroke patients [10]; importantly, miRNA could directly target and regulate proteins that were involved in stroke-related processes, such as plasminogen activator inhibitor-1 and MMP-9 [44]. Several miRNA such as miR-26a and miR145 exhibited neuroprotective properties by elevating the expression of interferon- (IFN-) beta (anti-inflammatory cytokine) [45]. In addition, the therapeutic potential of antagomirs (anti-miRNAs) has been confirmed in a number of *in vivo* models [46]. Hence, miRNAs are also a promising candidate for combating stroke. The latest research found that lncRNA-miRNA-mRNA constitutes an intricate regulatory network that participates in the pathophysiology of ischemic stroke and plays an important role in neuroprotection and postischemic recovery [47]. This work identified that TUG1, as a ceRNA for miR-3072-3p to target St8sia2, was a regulator of ischemic stroke.

Although it was previously reported that the number of cells with PSA- (synthesized by St8sia2-) NCAM marker was elevated in response to ischemia [33], the exact function of St8sia2 in stroke has not yet been completely clarified. In this research, we first determined an evident increase in St8sia2 expression in mouse brains under I/R as well as in N2A cells exposed to OGD/R and that elevated St8sia2 was accompanied by increased apoptosis. Previously, the enzymatic product of St8sia2, namely, PSA, was proposed to be responsible for polysialylation [48] that exerted proapoptotic effects in granulosa cells [49], which was in line with its proapoptotic property in the present study. It should also be noted that PSA regulate brain development and neural cell migration [50], which might be important for the repair of cerebral-ischemic injury. Hence, in the cerebral ischemia setting, St8sia2 might be a double-edged sword, and the adverse effects of St8sia2 might be ascribed to its interaction with other ischemia-promoting factors.

TUG1 was also recognized as a promoter of cardiomyocyte apoptosis through indirectly regulating proapoptotic KLF5 via miR-9a-5p [51]; in this study, we also found a positive correlation between TUG1 and ischemia-induced cerebral apoptosis. Moreover, we observed an elevated TUG1 expression that coincided with aggravated ischemic injury after I/R treatment, which was later reversed by TUG1 knockdown; these results also agreed with the observations of TUG1-promoted myocardial infarction [51]. Collectively, we discovered that TUG1 could also aggravate the cerebral ischemic injury and induce apoptosis in experimental models, in addition to its ischemia-promoting role in cardiomyocyte that was already established [51]. Li et al. [52] demonstrated that inhibiting the expression of TUG1 could protect mouse astrocyte cells and reverse the decrease in growth viability and increasing apoptosis of mouse astrocyte cells caused by OGD/R stimulation.

Intriguingly, the elevation of St8sia2 after the induction of ischemic injury coincided with increased TUG1/decreased miR-3072-3p expression. Subsequently, the binding of miR-3072-3p to both TUG1 and St8sia2 was confirmed by LRGAs. Although the exact role of miR-3072-3p was not previously reported, due to its inhibitory effect on ischemic apoptosis (confirmed by miR-3072-3p knockdown alone), we propose that miR-3072-3p not only serve as a bridge between TUG1 and St8sia2 but also alleviate the ischemic injury. In addition, previous study [53] has found that TUG1 aggravated cerebral ischemia and reperfusion injury by sponging miR-493-3p/miR-410-3p. This suggested that TUG1 might obtain the same mechanism by sponging miR-3072-3p.

Notably, inhibition of TUG1/St8sia2 or overexpression of miR-3072-3p partially antagonized the ischemic injury in several aspects including reduced infarct area, decreased neurologic deficit score, and attenuated apoptosis. Specifically, knockdown of St8sia2 alone exhibited an anti-ischemic effect similar to that induced by TUG1 inhibition/miR-3072-3p overexpression, suggesting that the effect of TUG1-miR-3072-3p/St8sia2 axis might converge on St8sia2.

However, the mechanism of the effect of the TUG1-miR-3072-3p/St8sia2 axis still needs to be further studied. There might be another signaling pathway involved with the TUG1-miR-3072-3p/St8sia2 axis to coprotect cerebral ischemia/reperfusion injury. Our prospect is to deeply investigate the TUG1-miR-3072-3p/St8sia2 axis in cerebral ischemia/reperfusion injury and apply it into clinical aspect which hopefully is a potential choice for the diagnosis/treatment of ischemic stroke.

## 5. Conclusion

In summary, the regulatory cascade identified in the current study provides a novel perspective for understanding the molecular mechanism underlying the pathogenies of ischemic stroke, as well as providing a theoretical basis for the diagnosis/treatment of ischemic stroke.

## Figures and Tables

**Figure 1:** TUG1 and St8sia2 were upregulated and accompanied by reduced miR-3072-3p level following *in vitro* and *in vivo* ischemic injuries. (a–g) C57BL/6J mice were subjected to MCAO/R (1.5 h/24 h) or sham operation. (a) Images of brain sections (underwent sham operation or I/R treatment) with TTC staining, the infarction zones were stained white. (b) Cerebral infarct ratio quantified by ImageJ. (c) Neurological deficit scores; the higher score represents more severe neurological deficit. (d) Expression of cerebral TUG1 at the transcript level in response to I/R was quantitated by Q-PCR. (e) Expression of cerebral miR-3072-3p at the transcript level in response to I/R was quantitated by Q-PCR. (f) Expression of cerebral St8sia2 at the transcript level in response to I/R was quantitated by Q-PCR. (g) Cerebral Bcl-2 and Bax levels in response to I/R were measured by western blot analysis. (h–m) N2A cells were subjected to OGD/R (4 h/24 h). Untreated cells were regarded as control. (h) Cellular Bcl-2 and Bax levels in response to oxygen glucose deprivation/reoxygenation were measured by western blot analysis. (i) Representative cell images of the TUNEL staining (scale bar = 25 *μ*m), N2A cells with excessive DNA damage were stained with red (TUNEL), whereas the blue counterstaining (DAPI) localized the nuclei. (j) Cell apoptosis percentage was quantified based on TUNEL-positive cells. (k–m) Expression of cerebral TUG1 at the transcript level in response to oxygen glucose deprivation/reoxygenation was quantitated by Q-PCR. (l) Expression of cerebral miR-3072-3p at the transcript level in response to oxygen glucose deprivation/reoxygenation was quantitated by Q-PCR. (m) Expression of cerebral St8sia2 at the transcript level in response to oxygen glucose deprivation/reoxygenation was quantitated by Q-PCR. ^∗^*P* < 0.05, ^∗∗^*P* < 0.01, and ^∗∗∗^*P* < 0.001. Sham: sham-operated animals; I/R: MCAO-induced ischemia/reperfusion group; control: untreated cells; OGD/R: oxygen glucose deprivation/reoxygenation group.

**Figure 2:** TUG1 knockdown attenuated *in vivo* ischemic injuries, accompanied by reduced St8sia2 and elevated miR-3072-3p levels. (a) Images of brain sections (underwent sham operation or I/R treatment combined with si-TUG1 or si-NC) with TTC staining, the infarction zones were stained white. (b) Cerebral infarct ratio quantified by ImageJ. (c) Neurological deficit scores; the higher score represents more severe neurological deficit. (d) Expression of cerebral TUG1, miR-3072-3p, and St8sia2 at the transcript level in response to I/R combined with si-NC or si-TUG1 was quantitated by Q-PCR. (e) Expression of cerebral miR-3072-3p at the transcript level in response to I/R combined with si-NC or si-TUG1 was quantitated by Q-PCR. (f) Expression of cerebral St8sia2 at the transcript level in response to I/R combined with si-NC or si-TUG1 was quantitated by Q-PCR. (g) Cerebral Bcl-2/Bax protein levels in response to I/R combined with si-NC or si-TUG1 were measured by western blot analysis. (h) Cerebral St8sia2 protein levels in response to I/R combined with si-NC or si-TUG1 were measured by western blot analysis. (i) Representative tissue images of the TUNEL staining (scale bar = 25 *μ*m), cerebral cells with excessive DNA damage were stained with green (TUNEL), whereas the blue counterstaining (DAPI) localized the nuclei. (j) Cell apoptosis percentage was quantified based on TUNEL-positive cells. (k) IHC staining intensity of St8sia2 was quantified by ImageJ. (l) Representative IHC image for St8sia2 in brain tissues that underwent I/R treatment combined with si-NC or si-TUG1. ^∗^*P* < 0.05, ^∗∗^*P* < 0.01, and ^∗∗∗^*P* < 0.001.

**Figure 3:** Forced overexpression of TUG1 resulted in ischemic-vulnerable phenotype of N2A cells opposite to that induced by TUG1 knockdown. (a–c) Expression of cerebral TUG1 at the transcript level in N2A cells underwent TUG1 overexpression (pc-DNA3.1-TUG1) or TUG1 knockdown (si-TUG1) was quantitated by Q-PCR. (b) Expression of cerebral miR-3072-3p at the transcript level in N2A cells (c) Expression of cerebral St8sia2 at the transcript level in N2A cells. (d, e) Bcl-2/Bax cell apoptosis percentage was quantified based on TUNEL-positive cells. (f) Representative cell images of the TUNEL staining (scale bar = 25 *μ*m), N2A cells with excessive DNA damage were stained with red (TUNEL), whereas the blue counterstaining (DAPI) localized the nuclei. (g) Protein levels in response to TUG1 overexpression/knockdown were measured by western blot analysis. ^∗^*P* < 0.05, ^∗∗^*P* < 0.01, and ^∗∗∗^*P* < 0.001.

**Figure 4:** miR-3072-3p directly binds to St8sia2 and regulates St8sia2 expression. (a) The sequence of wild-type St8sia2 (St8sia2-WT) and the mutant St8sia2 with mutations at the predicted miR-3072-3p binding site (St8sia2-MUT). (b, c) The luciferase reporter vector carrying St8sia2-WT or St8sia2-MUT or the empty vector was cotransfected into N2A cells with miR-3072-3p mimic or mimic-NC, the relative luciferase activity was detected 48 h after transfection. (c) The luciferase reporter vector carrying St8sia2-WT or St8sia2-MUT or the empty vector was cotransfected into N2A cells with miR-3072-3p inhibitor or inhibitor-NC, the relative luciferase activity was detected 48 h after transfection. (d) The direct interaction between St8sia2 and miR-3072-3p was confirmed by RNA immunoprecipitation assay after being transfected with miR-3072-3p mimic or mimic-NC for 48 h. (e) Expression of St8sia2 in N2A cells at the transcript level was measured 48 h post miR-3072-3p inhibitor transfection. (f) Expression of St8sia2 in N2A cells at the transcript level was measured 48 h post miR-3072-3p mimic transfection. Untransfected cells were defined as control (control). ^∗^*P* < 0.05, ^∗∗^*P* < 0.01, and ^∗∗∗^*P* < 0.001.

**Figure 5:** miR-3072-3p overexpression protects against I/R-induced ischemic injury in brain tissues. (a) Images of brain sections (underwent sham operation or I/R treatment combined with miR-3072 mimic or mimic-NC) with TTC staining, the infarction zones were stained white. (b) Cerebral infarct ratio quantified by ImageJ. (c) Neurological deficit scores; the higher score represents more severe neurological deficit. (d) Expression of cerebral miR-3072-3p at the transcript level in response to I/R combined with miR-3072 mimic or mimic-NC was quantitated by Q-PCR. (e) Expression of cerebral St8sia2 at the transcript level in response to I/R combined with miR-3072 mimic or mimic-NC was quantitated by Q-PCR. (f) Cerebral St8sia2 protein levels in response to I/R combined with si-NC or si-TUG1 were measured by western blot analysis. (g) Cerebral Bcl-2/Bax protein levels in response to I/R combined with si-NC or si-TUG1 were measured by western blot analysis. (h) Representative tissue images of the TUNEL staining (scale bar = 25 *μ*m), cerebral cells with excessive DNA damage were stained with green (TUNEL), whereas the blue counterstaining (DAPI) localized the nuclei. (i) Cell apoptosis percentage was quantified based on TUNEL-positive cells. ^∗^*P* < 0.05, ^∗∗^*P* < 0.01, and ^∗∗∗^*P* < 0.001.

**Figure 6:** miR-3072-3p overexpression protects against OGD/R-induced ischemic injury in N2A cells. (a, b) Expression of cellular miR-3072-3p and St8sia2 at the transcript level after the treatment with miR-3072-3p mimic or inhibitor was quantitated by Q-PCR. (c) Bar plot of cellular St8sia2 at the protein level after treatment was measured by western blot. (d) Expression of cellular St8sia2 at the protein level after treatment was measured by western blot and quantified. (e) Representative cell images of the TUNEL staining (scale bar = 25 *μ*m), N2A cells with excessive DNA damage were stained with red (TUNEL), whereas the blue counterstaining (DAPI) localized the nuclei. (f) Cell apoptosis percentage was quantified based on TUNEL-positive cells. (g) Alteration of Bcl2/Bax expression in N2A cells at the protein level after the treatment of miR-3072-3p mimic/inhibitor. ^∗^*P* < 0.05, ^∗∗^*P* < 0.01, and ^∗∗∗^*P* < 0.001.

**Figure 7:** TUG1 acts as a ceRNA for miR-3072-3p to target St8sia2. (a) The sequence of wild-type TUG1 (TUG1-WT) and the mutant TUG1 with mutations at the predicted miR-3072-3p binding site (TUG1-MUT). (b) The luciferase reporter vector carrying TUG1-WT or TUG1-MUT or the empty vector was cotransfected into N2A cells with miR-3072-3p mimic or mimic-NC; the relative luciferase activity was detected 48 h after transfection. (c) The luciferase reporter vector carrying St8sia2-WT or St8sia2-MUT or the empty vector was cotransfected into N2A cells with pcDNA3.1-TUG1 (along with the corresponding control); the relative luciferase activity was detected 48 h after transfection. (d) The luciferase reporter vector carrying St8sia2-WT or St8sia2-MUT or the empty vector was cotransfected into N2A cells with si-TUG1 (along with the corresponding control); the relative luciferase activity was detected 48 h after transfection. ^∗^*P* < 0.05.

**Figure 8:** St8sia2 might account for the regulatory effects of the TUG1-miR-3072-3p-St8sia2 axis in both *in vivo* and *in vitro* settings. (a) Images of brain sections (underwent sham operation or I/R treatment combined with si-St8sia2 or si-NC) with TTC staining, the infarction zones were stained white. (b) Cerebral infarct ratio quantified by ImageJ. (c) Neurological deficit scores; the higher score represents more severe neurological deficit. (d) Expression of cerebral St8sia2 at the transcript level in response to I/R combined with si-St8sia2 mimic or si-NC was quantitated by Q-PCR. (e) Cerebral St8sia2 protein levels in response to I/R combined with si-St8sia2 mimic or si-NC treatment were measured by western blot analysis. (f) Cerebral Bcl-2/Bax protein levels. (g) Alteration of St8sia2 expression in N2A at the protein level after the treatment of si-St8sia2 mimic or si-NC. (h) Alteration of Bcl2/Bax expression in N2A at the protein level after the treatment of si-St8sia2 mimic or si-NC. (i) Representative tissue images of the TUNEL staining (scale bar = 50 *μ*m), N2A cells with excessive DNA damage were, respectively, stained with green/red (TUNEL), whereas the blue counterstaining (DAPI) localized the nuclei. (j) Representative tissue images of the TUNEL staining (scale bar = 50 *μ*m) of cerebral cells. (k) Cell apoptosis percentage of N2A cells was quantified based on TUNEL-positive cells. (l) Cell apoptosis percentage of cerebral cells was quantified based on TUNEL-positive cells. ^∗^*P* < 0.05, ^∗∗^*P* < 0.01, and ^∗∗∗^*P* < 0.001.

**Table 1:** The primer sequences.

Subjects	The primer sequences
TUG1	Forward: 5′-TTCCTACCACCTTACTACTGACG-3′
	Reverse: 5′-GGAGGTAAAGGCCACATC-3′

miR-3072-3p	TGCCCCC TCCAGGAAGC CTTCTT

St8sia2	Forward: 5′-GACATAACCAGACGCTCTCTCT-3′
	Reverse: 5′-ACGATGGCACAAGTCCCAAA-3′

U6	Forward: 5′-GACTGCGCAAGGATGACAC-3′
	Reverse: 5′-CAGTGCGTGTCGTGGAGTC-3′

*β*-Actin	Forward: 5′-TTGCCGACAGGATGCAGAA-3′
	Reverse: 5′-GCCGATCCACACGGAGTACT-3′

## Data Availability

The labeled dataset used to support the findings of this study are available from the corresponding author upon request.
